RETRACTED

# Impact of donors’ financial fairness perception on donation intention in nonprofit organizations after COVID-19 outbreak

**DOI:** 10.1371/journal.pone.0251991

**Published:** 2021-06-09

**Authors:** Xia Li, Linyan Feng

**Affiliations:** 1 Accounting School, Anhui University of Finance and Economics, Bengbu, Anhui, China; 2 College of Business Administration, Anhui University of Finance and Economics, Bengbu, Anhui, China; Qingdao University, CHINA

## Abstract

Based on the investigation of financial fairness perception and donation intention of individual donors in non-profit organizations (NPOs), this paper uses structural equation model to analyze the impact of individual donors’ financial fairness perception on donation intention. The results show that individual donors’ perceptions on financial result fairness, financial procedure fairness and financial information fairness all have positive impact on donation intention; among which the perception on financial result fairness only has direct impact on individual donation intention, while the perceptions on financial procedure fairness and financial information fairness have direct and indirect impact on individual donation intention.

## Introduction

At the turn of 2020 and 2019, the turbulent coming and rapid spread of COVID-19 have seriously affected the normal life of people and caused great losses to economy and society, while the whole country is united to fight the epidemic, and the non-profit organizations (NPOs) have also actively involved in the fight, fulfilled their social responsibilities and made great contributions to the fight against the epidemic. The donation information issued by NPOs shows the important role of individual donation. Individual charitable donation as an important factor to promote social fairness and justice and maintain social harmony and stability also has outstanding performance in public emergencies such as epidemic situation. As of March 15, 2020, the data of some individual donations in China are shown in Table 1. As an important driving factor of donation behavior, individual donation intention acts on individual donation motivation [1], and directly affects individual donation behavior, which is affected by various perceptions and emotional factors of donors, such as their moral identity [2], perceived recipient benefit [3], etc. The donors’ subjective perception of donation-related issues has a direct impact on their psychology and behavior, which is related to the amount, frequency and direction of donation, as shown in Fig 1. Therefore, the research on this problem has important theoretical value and practical significance.

**Fig 1:** The impact of the donor’s personal perception on the donation.

RETRACTED

**Table 1:** Some individual donations in China. Unit: ten thousand yuan.

personal data	Yi-ming Zhang	Employees of ICBC	Employees of CCB	Wanda employees	Hai-hong Zhou	Qi-hu Qian
Donation amount (RMB)	10000	6100	5660	1600	1000	650

Data sources:https://m.jiemian.com/article/3933806.html(Interface news net).

• As an intermediary connecting donors and charitable beneficiaries, NPO will affect individual donors’ donation intention by its various situations, especially the financial position of organizations related to charitable funds. The reasonable allocation, effective use, reasonable financial procedure, transparent financial information and other aspects of charitable funds in NPOs are all concerned by donors, especially in the case of life-threatening epidemic, which are served as an important part of financial fairness to reflect the requirements of NPO stakeholders from different financial links. Financial fairness of NPO refers to the satisfaction of various stakeholders’ interests and requirements by reasonable resource allocation of NPOs, which is implemented in the whole process of funds movement and reflected in all aspects of financial activities and financial relations, Including organization fund raising, use and so on. It is the concrete embodiment of equity in non-profit finance, including equity of financial results, equity of financial procedures and equity of financial information, which respectively reflect the reasonable degree of the use result, use procedure and relevant financial information disclosure of financial funds in non-profit organizations. Financial fairness of NPO requires the organization to comprehensively consider the interests of stakeholders and try to be relatively fair in financial decisions, so as to realize the unity of economic and social benefits, and better fulfill the public accountability. Financial fairness of NPO includes objective and subjective levels, among which the former is realized by financial governance and management, while the latter is reflected in the subjective perception of stakeholders, as shown in Fig 2. And donors as the core stakeholders of the organization will directly affect donation intention by their financial fairness perception, thus affecting donation behavior.

**Fig 2:** The financial fairness frame of NPOs.

In the period of COVID-19, during the allocation of donated funds and goods by some NPOs, the phenomena of unfair distribution, overstocking of goods, low distribution efficiency, and delayed release of financial information, occurred in the links of goods acceptance, storage and distribution, have affected the process of epidemic prevention, seriously damaged the rights and interests of NPO stakeholders, and hit donors’ donation intention. Then, under the epidemic situation, how to better arrange resources to meet the relevant interests of donors, thus making them perceive financial fairness to enhance their donation intention? At present, the studies on influencing factors of individual donation intention of NPOs mainly focus on linear utility and emotional utility of donation, emotion, morality and prosocial behavior [4], accounting information of charitable organizations, and so on, while few scholars have deeply and systematically explored the impact of financial fairness perception on individual donation intention. Based on the investigation of financial fairness perception and donation intention of individual donors, this paper will explore the impact path of financial fairness perception on donation intention, in the hope of providing a new perspective and feasible ideas for financial decisions of NPOs. The contributions of this paper are as follows: First, the analysis under the background of COVID-19 on individual donated funds of NPOs is conductive to enhancing the response ability of NPOs to make them play a better role in dealing with public health emergencies, so as to improve China’s overall emergency response ability; second, clarify the impact path of financial fairness perception on individual donation intention under the epidemic situation, and explore the impact mechanism of various dimensions of financial fairness on donation intention, so as to provide reference for the financing decisions of NPOs; third, based on the exploration on the relevance of three dimensions of financial fairness perception under the epidemic situation, analyze the psychology and behavior of individual donors as the core NPO stakeholders, so as to provide reference for the internal financial governance and external supervision of NPOs.

RETRACTED

The contents below are arranged as follows: Based on the theoretical analysis of financial fairness and donation intention of individual donors in NPO, the second part puts forward research hypothesis, with the construction of impact model of financial fairness perception on donation intention of individual donors in NPO under the COVID-19. The third part includes the analysis on research samples, introduction of measurement tools for financial fairness and donation intention, and the test on scale reliability and validity. The fourth part is the verification and analysis on model hypothesis. The fifth part is the analysis on conclusions to obtain the corresponding enlightenment. The final part is about the deficiency of this paper and the prospect of future research in this field.

## Hypotheses and model construction

### Hypotheses

Financial fairness perception as the subjective level of financial fairness in NPO refers to stakeholders’ subjective feeling on organizational financial fairness, with the emphasis on stakeholders’ fairness perception on financial matters related to their own rights and interests. With financial fairness perception mainly from the feelings on fund usage, fund safety, compliant and rational fund-use process, availability of relevant financial information and financial information quality, donors have no full ownership and revenue claim right of donated funds, but have the right to require NPO to manage and use the funds according to agreement, while some invisible agreements without the presentation in the form of explicit contracts cannot prevent the donors from exercising their rights. At the same time, donors’ right to know enables them to obtain the financial information on the use process and result of donated funds, while donors’ financial fairness perception also can be affected by the availability and quality of financial information. For the donors driven by altruistic motivation and personal reputation demand, their focus on financial matters of donated NPO will be different due to different donation motivations. Fund-raising activities, fund-using activities, financial information disclosure and other financial activities in non-profit organizations are interrelated with the core stakeholders. The organization needs the funds donated by the donors, and the donors’ donation decisions are also affected by the organization’s fund using and information disclosure, as shown in Fig 3.

**Fig 3:** The relationship of financial activities and donor behavior of NPOs.

According to different contents, financial fairness perception of individual donors can be divided into perceptions on financial result fairness, financial procedure fairness and financial information fairness. Perceived financial result fairness refers to donors’ perception of satisfaction with the use of donated funds, which is directly related to donors’ donation expectations. Financial procedure perception refers to the donor’s satisfaction perception of the use of donated funds, which directly determines the use effect of funds. Perception of financial information fairness refers to the degree of perception of donors to the financial information disclosure of the recipient non-profit organizations. Under the epidemic situation, financial result fairness mainly focuses on the allocation of donated funds to the required areas, the achievement of expected goal in the use effect of funds, and the efficiency of organizing the fight against the epidemic. Financial procedure fairness mainly focuses on the use of funds according to relevant regulations and agreements, the good implementation of financial accounting system by NPO, the transparent source and use-process of donated funds for the epidemic, and the existence of black-box operation. Financial information fairness mainly focuses on the donated NPO’s concern on donors’ ideas about the use of funds, their provision of information about the use of funds, the procedure and process of use, and the reliability of the provided information.

RETRACTED

Facing the epidemic situation, the three dimensions of individual donors’ financial fairness perception do not exist in isolation, but jointly affect the psychology and behavior of donors on the basis of interrelations and mutual influence. The relationship of the three dimensions is shown as Fig 4. In order to timely provide donors with high-quality financial information, NPOs must do a good job in daily financial management by allocating the funds strictly according to regulations, making the funds management transparent, closely concerning on donors’ requirements for the use of funds, and rationally and effectively using the funds, thus only in this way can it better meet the rights and interests of donors and improve the financial management level of organization itself. Therefore, financial information fairness can play a powerful role in promoting the optimization of fund use-process and the improvement of utilization efficiency. On the other hand, in order to realize the efficient allocation of funds for the prevention of epidemic and fulfill donors’ wishes, NPOs must pay attention to the process management and reasonably arrange the use and distribution of funds, so as to promote the idealization of results with the standardization of process.

**Fig 4:** The relationship of three dimensions of financial fairness.

The following hypotheses are made according to the above analysis:

H1: Under the epidemic situation, financial information fairness perception of individual donors in NPO positively affects financial procedure fairness perception.
H2: Under the epidemic situation, financial information fairness perception of individual donors in NPO positively affects financial result fairness perception.
H3: Under the epidemic situation, financial procedure fairness perception of individual donors in NPO positively affects financial result fairness perception.

In common situation, donors’ behavior is consistent with their donation intention, except for the intention behavior related to compulsion and ignorance [5]. Under the epidemic situation, donation intention will drive the donation behavior of individual donors, which is often affected by factors such as the importance perception on public welfare matters. The impact on normal life during the epidemic has forced people to pay special attention to public welfare matters, especially in the face of possible anxiety caused by the epidemic. At this time, the closer relationship between NPO’s financial behavior and donors’ charity heart makes donors’ perception on charitable funds particularly sensitive, and their fairness perception on NPO’s financial decisions is more likely to affect their donation intention and donation behavior.

RETRACTED

The objectives of information disclosure by NPOs must meet the information needs of organizational external stakeholders, and the relationship maintenance and management of individual donors as an important link in the fund chain are an important task for NPO to disclose financial information for their social responsibility [6]. Under the epidemic situation, individuals’ understanding on the use of charitable funds is very important for the formation of donator’s attitude towards donation. NPOs should disclose the origin and development of epidemic funds in time, so as to make donors fully feel the role of their love in the fight against the epidemic, sense the satisfaction and happiness, and stimulate their donation intention.

Based on the effective utilization of charitable funds in the process of epidemic relief, the understanding on the process of funds movement by available financial information can make donors personally experience their help to recipients and contribution to society, with the sense of receiving gratitude feedback that will increase donors’ perception of social value and constantly promote their donation intention [7]. Many donors are unable to accurately see the exact use of funds they donated from the information issued by NPO, but they can see the information about operation procedure and operation results of similar funds. The more transparent the allocation of charitable funds donated to an organization, the more the operation process can reflect the strictness and preciseness of handling affairs according to regulations, the more the donors believe their funds can be properly arranged, and the higher their donation intention. The achievement of donors’ expected effect by the donated funds of NPO in the usage area and effect will stimulate more continuous donation.

The following hypotheses are obtained according to the above analysis:

H4: Under the epidemic situation, financial result fairness perception of individual donors in NPO positively affects their donation intention.
H5: Under the epidemic situation, financial procedure fairness perception of individual donors in NPO positively affects their donation intention.
H6: Under the epidemic situation, financial information fairness perception of individual donors in NPO positively affects their donation intention.

RETRACTED

### Model construction

According to the above hypotheses, it can obtain the models for financial fairness perception and donation intention of individual donors in NPO under the epidemic situation, as shown in Fig 5.

**Fig 5:** Models for financial fairness perception and donation intention of individual donors in NPO.

## Data acquisition and measurement index

### Research samples

• During the period of COVID-19, the questionnaires were distributed on February 28, 2020 to the people with donation experience for data acquisition, and as of March 4, 376 valid questionnaires were collected, with the basic information of all valid samples shown in Table 2. The questionnaire was released through the Questionnaire Star platform.

**Table 2:** Statistics for basic characteristics of samples.

Items	State Variable	Number of people(pcs)	Percentage (%)	Items	State Variable	Number of people(pcs)	Percentage (%)
Gender	male	126	33.51	Age	≤20	32	8.51
	female	250	66.49		21–30	163	43.35
Education degree	master or above	213	56.65		31–40	87	23.14
	undergraduate	152	40.43		41–50	64	17.02
	junior college student	7	1.86		51–60	29	7.71
	others	4	1.07		>60	1	0.27
Politics status	Communist Party of China	185	49.2	Position	intern	143	38.03
	league member	114	30.32		on job	218	57.98
	democratic parties	11	2.93		unemployed	14	3.72
	the masses	66	17.55		retired	1	0.27
Annual household income	≤30000	47	12.5	Personal monthly income	<1000	125	33.24
	30000–50000	44	11.7		1000–3000	41	10.9
	50000–80000	46	12.23		3000–5000	39	10.37
	80000–100000	54	14.36		5000–8000	94	25
	100000–200000	110	29.26		8000–10000	31	8.24
	>200000	75	19.95		>10000	46	12.23
Be religious or not	yes	19	5.05	Residential location	Hubei province	11	2.93
	no	357	94.95		not Hubei province	265	97.07

Among the respondents with donation to COVID-19, 14.95% of them donated less than 100 yuan, 55.34% donated between 100–499 yuan, 5.34% donated between 500 and 999, and 4.37% donated more than 1,000 yuan.

### Measurement index

Combined with the epidemic situation, the individual donors’ financial fairness scale [8] is used to measure individual financial fairness during the epidemic after the adjustment of measurement items, which originates from the fairness perception scales of [9–14], and constitutes of three dimensions, that is, financial result fairness, financial procedure fairness and financial information fairness, originally having 2, 3 and 3 items respectively. When in use, in order to better measure the various dimensions of individual donors’ financial fairness, the measurement items of financial result fairness that "the use area and effect of funds can achieve your expected goal" is divided into two items: "the use area of funds can achieve your expected goal" and "the use effect of funds can achieve your expected goal". The item of financial procedure fairness that "the source and use of organizational funds are open and transparent" is divided into two items: "the source of organizational funds is open and transparent" and "the use of organizational funds is open and transparent". Therefore, the final financial fairness scale includes 10 items in total, 3 for financial result fairness, 4 for financial procedure fairness and 3 for financial information fairness. Then the items in the above scale are adjusted to more accurately reflect the impact of the epidemic situation, for example, the donated organizations and the use of donated funds in each item are specified as the organizations donated by respondents during the epidemic and the corresponding use of funds, so as to better analyze the financial fairness perception of donors. Experts in the field of finance and NPOs from both theoretical and practical fields are also invited to analyze each item according to the research purpose and research object, thus the financial fairness scale used in the questionnaire is finally determined. The financial result fairness, financial procedure fairness and financial information fairness scale is shown as Tables 3–5.

RETRACTED

**Table 3:** Financial result fairness scale.

dimension	symbol	item
DJ	DJ1	The use area of funds can achieve your expected goal.
	DJ2	The use effect of funds can achieve your expected goal.
	DJ3	The money you donate to a nonprofit is used more effectively than any other organization in the same industry during the epidemic.

**Table 4:** Financial procedure fairness scale.

dimension	symbol	item
PJ	PJ1	The recipient non-profit organization can use the funds in accordance with relevant regulations and agreements.
	PJ2	The source of organizational funds is open and transparent.
	PJ3	The use of organizational funds is open and transparent.
	PJ4	The recipient NPO is able to implement the relevant financial and accounting systems well.

**Table 5:** Financial information fairness scale.

dimension	symbol	item
IJ	IJ1	The recipient nonprofit can provide me with detailed information about how the money will be used.
	IJ2	The recipient nonprofit can provide me with information about the procedures and processes for using the funds.
	IJ3	The recipient nonprofit cared about my thoughts on how to use the money and was able to communicate with me proactively.

The results of exploratory factor analysis and test on the financial fairness scale show that the KMO value of the scale is 0.880, the explained total variance is 80.053%, the factor loads are all greater than 0.7, and the α coefficients of financial result fairness, financial procedure fairness and financial information fairness are 0.831, 0.912 and 0.909, respectively, with good reliability and validity.

RETRACTED

The measurement on individual donation intention uses the scale used by [15] including four items, shown as Table 6.

**Table 6:** Individual donation intention scale.

dimension	symbol	item
DW	DW1	You are willing to donate to the NPO of your choice.
	DW2	You are still willing to donate to the NPO of your choice next time.
	DW3	You will not stop donating to the NPO that you have donated.
	DW4	You are willing to recommend others to donate to the NPO of your choice.

The KOM value of the scale is 0.770, with the coefficient of 0.953, explained total variance of 87.78%, and good reliability and validity. Due to the impact of donors’ personal characteristics on their donation intention, based on the combination of previous research achievements and the consideration of current situation, the gender, age, personal income, education degree, political status, religious belief and other factors are used as control variables [3, 16].

## Data analysis

### Validity and reliability

The model is conducted with exploratory factor analysis and confirmatory factor analysis by using SPSS21.0 and AMOS21.0, with the results shown in Tables 7 and 8, while the KMO value is 0.880, greater than 0.7, the factor load of each item is greater than 0.7, CR value of each factor is higher than 0.8, AVE of each latent variable is greater than 0.6, and all factors have good convergence validity. The square root of AVE of all latent variables is greater than the correlation coefficient between each latent variable and other latent variables, with the good discriminant validity between latent variables. In addition, confirmatory factor analysis shows that the good fitting between most fit indicators of model and data (X^2^/DF = 1.911, RMSEA = 0.067, RMR = 0.067, CFI = 0.977 and TLI = 0.971) indicates the good construct validity of model.

**Table 7:** Confirmatory factor analysis.

Dimensionality	Test Item	Factor Loading	CR	Reliability
Distribution Justice (DJ)	DJ1	0.832^a^	0.8378	0.831
	DJ2	0.839***		
	DJ3	0.711***		
Procedural Justice (PJ)	PJ1	0.777***	0.9136	0.912
	PJ2	0.898***		
	PJ3	0.893***		
	PJ4	0.835^a^		
Information Justice (IJ)	IJ1	0.955***	0.9185	0.909
	IJ2	0.954***		
	IJ4	0.744^a^		
Donation willingness (DW)	DW1	0.848^a^	0.943	0.953
	DW2	0.861***		
	DW3	0.949***		
	DW4	0.928***		

Notes:

^a^ represents the item whose normalization factor load defaults to 1, and

*** represents that the factor load is significant at the significance level of 0.01.

RETRACTED

**Table 8:** Correlation coefficient of latent variables and AVE value.

	**AVE**	**DJ**	**PJ**	**IJ**	**DW**
DJ	0.6339	0.7962			
PJ	0.7262	0.737	0.8522		
IJ	0.7919	0.690	0.555	0.8899	
DW	0.8056	0.709	0.659	0.616	0.8976

Notes: The data in diagonal bold represents the square root value of AVE of each factor.

### Path analysis

The analysis results by AM0S21.0 show that χ^2^ /df = 1.911 (p < 0.001), TLI = 0.971, CFI = 0.977, and GFI = 0.920, indicating the good goodness-of-fit of model, as shown in Table 9.

**Table 9:** Goodness-of-fit index of model.

	χ^2^ /df	IFI	TLI	GFI	CFI	RMSEA	RMR
Standard Values	≤3	>0.9	>0.9	>0.9	>0.9	<0.08	<0.05
Model	1.911	0.978	0.971	0.920	0.977	0.067	0.067
Fitting Judgement	reach standard	reach standard	reach standard	reach standard	reach standard	reach standard	Sub- standard

In order to detect the statistical significance of the estimated parameters, the model path coefficient is conducted with statistical significance test, with the model path coefficient estimates shown in Table 10. The results show that under the epidemic situation, the financial information fairness perception of individual donors in NPO has the significantly positive impact on the perceptions of financial procedure fairness and financial result fairness, while financial procedure fairness perception has positive impact on financial result fairness perception, with the respective path coefficients of 0.555 (p<0.01), 0.406 (p<0.01) and 0.512 (p<0.01), thus H1, H2 and H3 are verified; under the epidemic situation, the perceptions on financial information fairness, financial procedure fairness and financial result fairness of individual donors in NPO have the significantly positive impact on their donation intention, with the respective path coefficients of 0.357 (p = 0.01), 0.257 (p = 0.02) and 0.217 (p = 0.06), thus H4, H5 and H6 are verified.

**Table 10:** Estimation on model path coefficient.

	Unnormalized Path Coefficient stimation	S.E.	C.R.	Significance	Coefficient Estimation
DW<−−−DJ	0.554	0.174	3.181	0.001**	0.357
DW<−−−IJ	0.336	0.123	2.742	0.006**	0.217
DW<−−−PJ	0.389	0.126	3.084	0.002**	0.275
DJ<−−−PJ	0.466	0.067	6.967	***	0.512
DJ<−−−IJ	0.405	0.072	5.618	***	0.406
PJ<−−−IJ	0.608	0.084	7.270	***	0.555

Notes:

*** represents that the factor load is significant at the significance level of 0.01.

## Conclusion and enlightenment

### Conclusions

As to the impact path of financial fairness perception on individual donation intention, under the epidemic situation, the perceptions on financial information fairness, financial procedure fairness and financial result fairness of individual donors in NPO have the positive impact on their donation intention, and jointly act on the donation psychology and behavior of donors. There are some differences in the impact path of the three dimensions of financial fairness perception on individual donors’ donation intention. The financial result fairness perception only has direct impact on individual donation intention, while the perceptions on financial procedure fairness and financial information fairness not only have direct impact on individual donation intention, but also have indirect impact on individual donation intention through financial result fairness perception. In addition, financial information fairness perception also has positive impact on donation intention through financial procedure fairness perception.

RETRACTED

As to the relationship between the three dimensions of financial fairness perception, the direct impact of financial information fairness perception of NPO on both financial procedure fairness perception and financial result fairness perception shows that financial information plays a fundamental role in financial fairness perception of individual donors, thus NPOs should pay attention to the various requirements of individual donors for financial information.

As to the impact of financial fairness perception on individual donation intention, among the direct impacts of the three dimensions of financial fairness perception of individual donors in NPO on donation intention, financial result fairness perception has the greatest impact, followed by financial procedure fairness perception, and finally the financial information fairness perception. Therefore, NPOs can first consider the financial result fairness with greatest impact when collecting donations.

As to the background of COVID-29, the author has studied the impact of financial fairness perception in NPO on individual donation intention during the normal situation (Li Xia et al., 2017), and the comparison between the applications of survey data in the same model in different situations shows that under the epidemic and normal situations, the impact paths of financial fairness perception of individual donors in NPO on donation intention are different. Under the normal situation, individual donors’ financial procedure fairness perception has no significant direct impact but has indirect impact on donation intention through financial result fairness perception, while the impact path of financial result fairness perception and financial procedure fairness perception is the same as that in the donation under the epidemic situation. In terms of impact degree, whether the donation is for the epidemic situation or not, financial result fairness has the greatest impact, and there is no difference in the path of mutual influence between the three dimensions of financial fairness. Under the epidemic situation, the significantly positive and direct impact of individual donors’ financial procedure fairness perception on donation intention may be related to the fuzziness of the use effect of donated funds and the difficulty of evaluation. In daily donation, the donors of NPOs will make clear the specific projects they donate and track the implementation of the corresponding projects in the donated organizations, while under the epidemic situation, except a small number of donors with targeted large-scale donation, most of the donated funds with shorter participation in the rescue relative to the daily projects often play a role together with other funds, thus the donors can only know the general use of donated funds, rather than accurately grasp the detailed information about the use of funds. According to the financial information issued by NPOs, most external stakeholders can only see the source and amount, the allocation and amount, but fail to know the corresponding relationship between corresponding relationship between sources and, so they will pay more attention to the fund operation process of NPOs, so as to investigate and infer the use effect of funds through the compliance and rationality of procedures. The equity of financial results, whether in the epidemic period or not, is the most direct embodiment of the utility available to donors, and directly affects the donor’s donation intention and behavior. Financial information, as a transmitter for donors to understand the effects and procedures of the use of donated funds, is the most important link between donors and recipient organizations, regardless of whether it is during the epidemic period, and has a significant impact on the psychology and behavior of donors. The consistency comparison of the influence path of financial equity on donation intention under different situations is shown as Tables 11 and 12.

RETRACTED

**Table 11:** Consistency comparison of significance.

item	Is the direct impact significance consistent in the two situations?
the impact of financial result fairness on willingness to donate	yes
the impact of financial procedure fairness on willingness to donate	no
the impact of financial information fairness on willingness to donate	yes

**Table 12:** Consistency comparison of the direct influence path.

item	Is the affect path consistent in the two situations?
the impact of financial result fairness on willingness to donate	yes
the impact of financial procedure fairness on willingness to donate	no
the impact of financial information fairness on willingness to donate	no

### Enlightenment

In the future, fighting against various epidemic is the common issue faced by human beings, and NPOs as an important force to continuously struggle on the anti-epidemic front is an important part of emergency response system, which can play a greater role in fighting against various epidemic by gathering the various social forces and making extensive use of social capital, thus NPOs with the bridging role in connecting the public and the relief objects will be selected by many people to help them fulfill wishes in epidemic prevention. On the other hand, the importance of individual donation in the source of funds for NPOs makes the study of individual donors’ financial fairness on donation intention have great significance for both donors and organizations.

Under the epidemic situation, in order to obtain more individual donated funds and improve the ability of epidemic prevention, NPOs must focus on donors’ donation intention and analyze their needs. Individual donors require NPOs to not only provide financial information and report the use area and effect of funds in time, but also provide reasonable and reliable information, with the hope of being concerned by and communicated with NPOs about donors’ ideas on the use of funds. However, the actual situation shows that the information disclosure system of NPOs is unable to meet the requirements of stakeholders for information [17, 18], and the information needs of donors are lack of strong institutional protection. In financing decision-making, NPOs should comprehensively consider donors’ needs for financial information, and disclose more information about individual donation decisions beyond the system provisions, so as to improve their attractiveness and obtain more funds. In the use of funds, NPOs should effectively use the donated goods and funds for the fight against the epidemic, and make the funds movement process normalized and transparent, so as to easily acquire the use effect of charitable funds by more external stakeholders, thus improving financial fairness perception and enhancing donation intention of donors.

After the outbreak, NPOs should focus on the psychological change of individual donors, enhance the incentive effect of the results of fund use on donors, and promote the unity of use efficiency and fairness of donated funds, so as to better perform the public accountability.

## Deficiency of this paper and prospect of future research

In this paper, the limitations caused by respondents including the overall higher educational background and the majority of donations within 500 yuan make the research results have poor explanatory power for donors with larger donation amount and other education background. The follow-up study should expand the sample range and conduct more in-depth analysis.

RETRACTED

Under the epidemic situation, the impact of individual donors’ financial fairness perception in NPOs on donation intention will develop towards the depth direction [19]. The different degree of economic development, the different extent of disaster and the different management system in each country and region will make the impact of individual donors’ financial fairness perception in NPOs on donation intention presented with different characteristics, which will be a possible research direction in this field in the future. In addition, the comparative study of the impact of individual donors’ financial fairness perception on donation intention under the epidemic or normal situations will also tend to refinement.

As the epidemic continues to spread, the fight against the epidemic cannot be slackened. Multi-party efforts should be pooled to fight the epidemic. In this context, how to better understand the donors, understand their donation psychology and behavior, will be an ongoing topic in the future.

## Ethics statement

This study (Impact of Donors’ Financial Fairness Perception on Donation Intention in Nonprofit Organizations after COVID-19 Outbreak) is not ethically sensitive and was carried out in accordance with national and institutional legal and ethical requirements. Written informed consent was obtained from all participants and interviewers confirmed that all participants had read the information leaflet before starting the interview. In this research all collected data would be only used for research anonymously, and this study falls outside the scope of Ethics. all collected data would be only used for research anonymously, therefore this study falls outside the scope of General Data Protection Regulation (GDPR) 2016.

## Supporting information

S1 Data (SAV)

S1 Questionnaire (PDF)

S2 Questionnaire (PDF)

## References

[1] GottfriedM. A., JohnsonE. L. Solicitation and Donation: An Econometric Evaluation of Alumni Gener-osity in Higher Education. International Journal of Educational Advancement.2006,6(7):268–281. doi: 10.1057/palgrave.ijea.2150034

[2] ReedA., AquinoK., LevyE. Moral Identity and Judgments of Charitable Behaviors. Journal of Marketing.2007,71(1):178–193. doi: 10.1509/jmkg.71.1.178

[3] AndorferVeronika A. and OtteGunnar. Do Contexts Matter for Willingness to Donate to Natural Disaster Relief? An Application of the Factorial Survey. Nonprofit and Voluntary Sector Quarterly. 2012,42(4):657–688. doi: 10.1177/0899764012440180

RETRACTED

[4] GoenkaShreyans, van OsseslaerStijn M J. Charities Can Increase the Effectiveness of Donation Appeals by Using a Morally Congruent Positive Emotion. Journal of Consumer Research.2019,46(4):774–790. doi: 10.1093/jcr/ucz012

[5] ZhaoF. F., DuL. Y., Research on influencing factors of employees’ donation intention based on organizational mobilization situation. Technology and Management. 2016, 2: 36–61.

[6] JohnM T, LindaM P. Financial Reporting Factors Affecting Donations to Charitable Organizations. Advances in Accounting. 2007, (23): 263–285. doi: 10.1016/S0882-6110(07)23010-X

[7] GrantA M, GinoF. A Little thanks goes a long way: explaining why gratitude expressions motivate prosocial behavior. Journal of Personality and Social Psychology.2010,98:946–955. doi: 10.1037/a0017935 20515249

[8] LiX., etc. Study on the Influence of perceived financial fairness of donors in non-profit organizations on their intention to donate. Journal of Shanghai University of Finance and Economics. 2017,19(5): 40–51.

[9] ColquittJ A. On the Dimensionality of Organizational Justice: A Construct Validation of a Measure. Journal of Applied Psychology. 2001,86(3):386–400. doi: 10.1037/0021-9010.86.3.386 11419799

[10] ThibautJ, WalkerL. Procedural Justice: A Psychological Analysis. Hillsdale, NJ: Lawrence. Erlbaum Associates.1975.

[11] LeventhalG S. The Distribution and Rewards and Resources in Groups and Organizations. In BerkowitzL & WalsterW, Advances in Experimental Social Psychology. New York: Plenum Press.1976,9:91–131. 10.1016/S0065-2601(08)60059-3

[12] LeventhalG S. What Should Be Done With Equity Theory?New Approaches to the Study of Fairness in Social Relationships. In GergenK J, GreenbergM S, WillisR H. Social Exchange: Advances in Theory and Research. New York: Plenum Press. 1980:27–55.

[13] BiesR J, MoagJ S. Interactional Justice: Communication Criteria of Fairness. In LewickiR J, SheppardB H, BazermanM H. Research on Negotiations in Organizations. Greenwich, CT: JAI Press.1986,1:43–55.

[14] ShapiroD L, ButtnerE H, BarryB. Explanations: What Factors Enhance Their Perceived Adequacy?.Organizational Behavior and Human Decision Processes. 1994,58:346–368. doi: 10.1006/obhd.1994.1041

[15] DuL. Y. etc. Research on the attractiveness of Individual donations from Non-profit organizations in China. Beijing: science press. 2012.4:182

[16] BrooksA C. Who Really Cares: The Surprising Truth About Compassionate Conservatism. New York: Basic Books, 2006.

RETRACTED

[17] KottaszR. How Should Charitable Organizations Motivate Young Professionals to Give Philanthropically. Journal of Nonprofit and Voluntary Sector Marketing. 2004,9(1):9–27. doi: 10.1002/nvsm.230

[18] AckermannK. Predisposed to Volunteer? Personality Traits and Different Forms of Volunteering. Nonprofit and Voluntary Sector Quarterly, 2019,48(6):1119–1142. doi: 10.1177/0899764019848484

[19] AlbouyJ., GalanJ.P., MaubissonL. Building Satisfaction and Loyalty During a Musical Benefit Event: A Consumer-Based approach. Nonprofit and Voluntary Sector Quarterly, 2019,48(6):1250–1271. doi: 10.1177/0899764019843341

